The article "Investigation of the hub genes and related mechanism in ovarian cancer via bioinformatics analysis" was retracted in 2015. Reasons: an official misconduct investigation; misconduct by an author; compromised peer review.

# Investigation of the hub genes and related mechanism in ovarian cancer via bioinformatics analysis

**DOI:** 10.1186/1757-2215-6-92

**Published:** 2013-12-17

**Authors:** Ling-jie Fu, Bing Wang

**Affiliations:** 1 Department of gynaecology and obstetrics, Shengjing hospital of China Medical University, No.36 Sanhao Street, Shenyang City 110004, China; 2 Ultrasound Department, Shengjing hospital of China Medical University, No.36 Sanhao Street, Shenyang City 110004, China

**Keywords:** Ovarian cancer, Protein-protein interaction network, Network module, Molecular mechanism

## Abstract

**Background:**

Ovarian cancer is a cancerous growth arising from the ovary.

**Objective:**

This study was aimed to explore the molecular mechanism of the development and progression of the ovarian cancer.

**Methods:**

We first identified the differentially expressed genes (DEGs) between the ovarian cancer samples and the healthy controls by analyzing the GSE14407 affymetrix microarray data, and then the functional enrichments of the DEGs were investigated. Furthermore, we constructed the protein-protein interaction network of the DEGs using the STRING online tools to find the genes which might play important roles in the progression of ovarian cancer. In addition, we performed the enrichment analysis to the PPI network.

**Results:**

Our study screened 659 DEGs, including 77 up- and 582 down-regulated genes. These DEGs were enriched in pathways such as Cell cycle, p53 signaling pathway, Pathways in cancer and Drug metabolism. *CCNE1*, *CCNB2* and *CYP3A5* were the significant genes identified from these pathways. Protein-protein interaction (PPI) network was constructed and network Module A was found closely associated with ovarian cancer. Hub nodes such as VEGFA, CALM1, BIRC5 and POLD1 were found in the PPI network. Module A was related to biological processes such as mitotic cell cycle, cell cycle, nuclear division, and pathways namely Cell cycle, Oocyte meiosis and p53 signaling pathway.

**Conclusions:**

It indicated that ovarian cancer was closely associated to the dysregulation of p53 signaling pathway, drug metabolism, tyrosine metabolism and cell cycle. Besides, we also predicted genes such as *CCNE1*, *CCNB2*, *CYP3A5* and *VEGFA* might be target genes for diagnosing the ovarian cancer.

## Introduction

Ovarian cancer which caused an estimated 22,430 new cases and 15,280 deaths in 2007 in the United States [1], is the leading cause of death from gynecologic malignancy [2]. Approximately 90% of primary malignant ovarian tumors are epithelial (carcinomas), which are from the ovarian surface epithelium (OSE) [3,4]. And ovarian epithelial tumors currently contains four major types of epithelial tumors (serous, endometrioid, clear cell, and mucinous) based entirely on tumor cell morphology. It is well known that the symptoms of it include bloating, pelvic pain, difficulty eating, frequent urination and so on. But it is difficult to diagnose ovarian cancer at its early stages (I/II) as its most symptoms are non-specific [5].

It is all known that tumors develop and progress are related to accumulated molecular genetic or genomic changes such as point mutation, gene amplification, deletion, and translocation [6]. For instance, *TP53* is mutated in 50% or more high-grade serous carcinomas [7]. Besides, it have been indicated that some tumor suppressor genes and oncogenes such as *BRCA1/2*, *PTEN*, and *PIK3CA* also mutated and accumulated in ovarian serous carcinomas [7-9]. Studies also demonstrated that the overexpression of *cyclin D1* has close relationship with low-grade ovarian carcinomas, which is consistent with the view that *cyclin D1* is a downstream target of active *MAPK* (mitogen-activated protein kinase) constitutively expressed in most low-grade ovarian tumors as a results of frequent activating mutations in *KRAS* (v-Ki-ras2 Kirsten rat sarcoma viral oncogene homolog) and *BRAF* (v-raf murine sarcoma viral oncogene homolog B1) [10-12]. In spite of the expanded efforts to study the genetic bases of ovarian cancer, the molecular mechanisms of the development and progression were still not clear.

In this study, we identified the differentially expressed genes (DEGs) between the ovarian cancer samples and the healthy controls. In addition, we used the DAVID (The Database for Annotation, Visualization and Integrated Discovery) to identify the significant KEGG pathways. Furthermore, we constructed protein-protein interaction networks to study and identify the target genes for diagnosing the ovarian cancer.

## Materials and methods

### Data source

The gene expression profiles of GSE14407 which was contributed by Bowen, N.J., *et al*. [13] were obtained from National Center of Biotechnology Information (NCBI) Gene Expression Omnibus (GEO) database (http://www.ncbi.nlm.nih.gov/geo/). The platform of the GPL570 ([HG-U133_Plus_2] Affymetrix Human Genome U133 Plus 2.0 Array) was applied in the expression array. The datasets available in this analysis contained 24 samples, including 12 ovarian cancer samples and 12 controls. These data (CEL form) and annotation files were downloaded for further analysis.

### Identification of DEGs

After obtaining the raw data, the RMA (Robust Multi-array Average) method [14] of the R software [15] was used to perform quartile data normalization, then the *t* test methods of the Limma package [16] was used to identify DEGs. Values of |log Fold Change (FC)| > 2.0 and p-value < 0.05 were selected as the cut-off criteria.

### The functional enrichment analysis of the DEGs

KEGG pathway database is a recognized and comprehensive database including all kinds of biochemistry pathways [17]. In this work, the KEGG database was applied to investigate the enrichment analysis of the DEGs to find the biochemistry pathways which might be involved in the occurrence and development of ovarian cancer. DAVID [18] was used to perform the KEGG pathway enrichment analysis with the p-value < 0.05 and gene count > 2.

### Protein-protein interaction network construction

Since proteins seldom perform their functions in isolation, it is important to understand the interaction of these proteins by studying larger functional groups of proteins [19]. In this study, the STRING online tools [20] were used to analyze the PPIs of the DEGs with the cut-off criterion of combined score > 0.4. The relationships of the nodes degree ≤ 5 were abandoned, then the Cytoscape software was used to construct the network [21]. Form the previous study, most obtained PPI networks obeyed the scale-free attribution [22]. So the node degree of the network was analyzed and used to obtain the hub protein in the PPI network. The node degree ≥30 were selected as the threshold.

### Network module analysis of the ovary cancer

The nodes and edges of the PPI network were so complicate that we need to conduct the enrichment analysis using the ClusterONE Cytoscape plug-in [23]. Minimum size >5 and minimum density < 0.05 were the parameters before running the ClusterONE to disclose the enriched functional modules of the PPI network. We also performed the GO (gene ontology) functional enrichment analysis of the module genes to analyze the gene function in the molecule level. Furthermore, the best enriched module was performed KEGG pathway enrichment analysis using DAVID [18].

## Results

### Identification of DEGs

Limma package in R was used to identify the DEGs between the ovarian cancer samples and the healthy controls. According to the cut-off criteria of |logFC| > 2.0 and p-value < 0.05, we finally gained 659 DEGs, including 77 up- and 582 down-regulated genes.

### KEGG pathways analysis

To gain further insights into the function of DEGs, DAVID were applied to identify the significant dysregulated KEGG pathways. The pathways obtained with p-value < 0.05 and gene count > 2 of the up- and down-regulated genes were showed in Table 1, respectively. According to the enrichment results, the up-regulated genes were significantly enriched in pathways such as Cell cycle and p53 signaling pathway; genes including *CCNE1* (cyclin E1) and *CCNB2* (cyclin B2) were identified in p53 signaling pathway. Besides, the down-regulated DEGs were enriched in Drug metabolism, Pathways in cancer and Tyrosine metabolism significantly. *CYP3A5* (cytochrome P450, family 3, subfamily A, polypeptide 5), *GSTM3* (glutathione S-transferase mu 3), *MAOA* (monoamine oxidase A) were the significant genes filtered out from the Drug metabolism pathway.

**Table 1:** The KEGG pathway of the DEGs

**Category**	**KEGG pathway term**	**Count**	**Genes**	**P-value**
Up-regulated DEGs	hsa00982 drug metabolism	8	CYP3A5, GSTM3, MAOA, …	0.004592
	hsa05200 pathways in cancer	21	WNT5A, BMP2, FGF9, …	0.006931
	hsa00980 metabolism of xenobiotics by cytochrome P450	7	AKR1C2, CYP3A5, GSTM3, …	0.015153
	hsa00350 tyrosine metabolism	6	MAOA, ALDH1A3, AOX1, …	0.015606
	hsa04610 complement and coagulation cascades	7	THBD, C3, CFH, TFPI, …	0.028328
	hsa00330 arginine and proline metabolism	6	GATM, MAOA, GLS, MAOB, …	0.032382
	hsa04510 focal adhesion	13	CAV2, CAV1, COL3A1, MET, …	0.038664
Down-regulated DEGs	hsa04110 cell cycle	7	CCNE1, CDKN2A, CCNB2, … BUB1B,	1.06E-05
	hsa04115 p53 signaling pathway	5	CCNE1, CDKN2A, CCNB2, …	1.78E-04
	hsa05200 pathways in cancer	7	CCNE1, FGF18, CDKN2A, …	0.002121
	hsa04114 oocyte meiosis	4	CCNE1, CCNB2, AURKA, …	0.011244

### PPI network construction

The STRING tool was used to get the PPI relationships of the DEGs. A total of 1241 PPI relationships were gained with the combined score > 0.4. After the nodes of degree ≤ 5 were filtered out, we finally built the network with 405 nodes and 1224 edges (Figure 1). The connectivity degree of each node of the PPI network was calculated and the results of some nodes were shown in the Table 2. The genes *VEGFA* (vascular endothelial growth factor A), *CALM1* (calmodulin 1), *BIRC5* (baculoviral IAP repeat containing 5), *POLD1* (polymerase-DNA directed, delta 1, catalytic subunit), *AURKA* (aurora kinase A), *CDT1* (chromatin licensing and DNA replication factor 1), *BUB1B* (BUB1 mitotic checkpoint serine/threonine kinase B) with high connectivity degree > 30 were selected as the hub nodes and might play important roles in the progression of ovarian cancer.

**Figure 1:** PPI network analysis of DEGs of ovarian cancer, node stand for the protein (gene), edge stand for the interaction of proteins.

**Table 2:** The statistical results of connectivity degrees of the PPI network

**Gene**	**Degree**
VEGFA	46
CALM1	38
BIRC5	36
POLD1	34
AURKA	34
CDT1	31
BUB1B	31

The gene in the table is the symbol of the protein (gene), degree stand for the connectivity degree of the gene.

### Module analysis

PPI network enrichment was one of the main methods to study and identify the functional proteins. In this study, there were 9 significant modules (p value <1 × 10^-3^) enriched by ClusterONE plug-in with the parameters of minimum size > 5 and minimum density < 0.05. And the most significant enrichments Module A (p = 1.000 × 10^-4^), Module B (p = 1.350 × 10^-7^) and Module C (p = 5.552 × 10^-7^) were showed in Figure 2. According to the Figure 2, it was obviously that Module A might be the best module as it has 30 nodes and 347 edges compared to Module B with 41 nodes and 69 edges as well as Module C with 45 nodes and 59 edges.

**Figure 2:** **The module of PPI network of ovarian cancer.** The **A**, **B**, **C** were respectively the modules with the lowest 3 p-value.

To further study the function changes in the course of tumor progression, we performed the GO functional annotation of genes in the Module A, Module B and Module C (Table 3). The GO enrichment scores of Module A, B and C were 17.28, 2.49 and 4.39, respectively. Therefore, Module A might be the most suitable module for further functional analysis. There were 30 genes in the Module A (Figure 2A), which were significantly enriched in the biological processes such as mitotic cell cycle, cell cycle and nuclear division. Then these genes were investigated by KEGG pathway enrichment analysis and the outcomes were shown in Table 4. The genes in this module were remarkable enriched in pathways such as Cell cycle, Oocyte meiosis, p53 signaling pathway, Pyrimidine metabolism and Purine metabolism. *CCNE1* and *CCNB2* were also the significant genes enriched in cell cycle pathway.

**Table 3:** The GO analysis of the three modules

**Category**	**Term**	**Description**	**Count**	**P value**
**Module A**	**Enrichment score: 17.28123992198**			
BP	GO:0000278	Mitotic cell cycle	18	1.21E-20
BP	GO:0007049	Cell cycle	21	6.99E-20
BP	GO:0022403	Cell cycle phase	18	8.21E-20
BP	GO:0022402	Cell cycle process	19	3.72E-19
BP	GO:0000279	M phase	16	5.88E-18
BP	GO:0000280	Nuclear division	14	6.30E-17
BP	GO:0007067	Mitosis	14	6.30E-17
BP	GO:0000087	M phase of mitotic cell cycle	14	7.98E-17
BP	GO:0048285	Organelle fission	14	1.07E-16
BP	GO:0051301	Cell division	14	3.01E-15
**Module B**	**Enrichment score: 2.48970202313**			
BP	GO:0009611	Response to wounding	8	5.04E-04
BP	GO:0050817	Coagulation	4	2.68E-03
BP	GO:0007596	Blood coagulation	4	2.68E-03
BP	GO:0007599	Hemostasis	4	3.16E-03
BP	GO:0050878	Regulation of body fluid levels	4	6.65E-03
**Module C**	**Enrichment score: 4.39218066431**			
MF	GO:0003700	Transcription factor activity	15	1.97E-07
MF	GO:0030528	Transcription regulator activity	18	1.97E-07
MF	GO:0043565	Sequence-specific DNA binding	12	6.00E-07
BP	GO:0006355	Regulation of transcription, DNA-dependent	19	7.70E-07
BP	GO:0051252	Regulation of RNA metabolic process	19	1.08E-06
BP	GO:0045449	Regulation of transcription	20	4.71E-05
MF	GO:0003677	DNA binding	18	8.11E-05
BP	GO:0006357	Regulation of transcription from	10	2.16E-04
		RNA polymerase II promoter		
BP	GO:0006350	Transcription	16	5.92E-04

Category stands for the GO function, BP stands for biological process, MF stands for molecule function, enrichment score stands for score of GO enrichment.

**Table 4:** The KEGG pathway of the genes in the Module A

**KEGG pathway term**	**Count**	**Genes**	**P-value**
hsa04110 cell cycle	5	CCNE1, CCNB2, BUB1B, TTK, PTTG1	1.00E-04
hsa04114 oocyte meiosis	4	CCNE1, CCNB2, AURKA, PTTG1	0.001432
hsa04115 p53 signaling pathway	3	CCNE1, CCNB2, RRM2	0.008966
hsa00240 pyrimidine metabolism	3	RRM2, POLD1, NME7	0.017022
hsa00230 purine metabolism	3	RRM2, POLD1, NME7	0.041398

## Discussion

Ovarian cancer is the seventh leading cause of cancer-related death in women [24]. It is difficult to detect this disease due to asymptomatic early-stage malignancy. Thus, most women although initially responsive, eventually develop and succumb to drug-resistant metastases [25]. So new drug targets and biomarkers that facilitate early detection of ovarian cancer are essentially needed and for further understanding the molecular pathogenesis.

In this study, we gained 659 DEGs including 77 up-regulated DEGs and 582 down-regulated DEGs upon gene expression profile of GSE14407. Most of these up-regulate DEGs were enriched in pathways of Cell cycle and p53 signaling pathway, while the down-regulated DEGs were significantly related to pathways such as Drug metabolism, Pathways in cancer and Tyrosine metabolism. Genes including *CCNE1*, *CCNB2*, *CYP3A5*, *GSTM3* and *MAOA* were significantly identified in these pathways.

It had indicated that p53 signaling pathway was one of the significant pathway enriched by up-regulated DEGs. P53 is a critical regulator of the response to DNA damage and oncogenic stress. It is associated with the growth, apoptosis and cell cycle arrest of cancer cells which can induce the inhibition of proliferation in cancer cells. Reles *et al*. also found that p53 alterations correlated significantly with resistance to platinum-based chemotherapy, early relapse, and shortened overall survival in ovarian cancer patients in univariate analysis [26]. Therefore, the dysregulation of p53 function is a frequent occurrence in human malignancies [27]. In this study, *CCNE1* and *CCNB2* of p53 signaling pathway were also up-regulated. *CCNE1* encodes a protein which belongs to the highly conserved cyclin family. It a regulatory subunit of CDK2 and its activity is required for cell cycle G1/S transition. A previous study indicated that its over-expression was important to growth and survival of ovarian cancer tumors [28]. *CCNB2* encodes the cyclin B2, which could bind to transforming growth factor beta RII and thus cyclin B2/cdc2 may play a key role in transforming growth factor beta-mediated cell cycle control. And it proved that *CCNB2* overexpressed in tumor tissue and may be used as a very reliable biomarker of lung adenocarcinoma [29]. So it indicated that p53 signaling pathway played important roles in ovarian cancer, and *CCNE1* and *CCNB2* might be potential diagnostic and therapeutic targets in ovarian cancer.

The down-regulate DEGs were significantly enriched in pathways such as Drug metabolism, Pathways in cancer and Tyrosine metabolism. The cytochromes P450 (CYPs) are key enzymes in cancer formation and cancer treatment as they regulate the metabolic activation of a large number of precarcinogens and participate in the inactivation and activation of anticancer drugs [30]. In addition, tyrosine is a non-essential amino acid that conjugates with corresponding tRNA forming Tyrosine-tRNA [31]. And targeted therapy for ovarian cancer with tyrosine kinase inhibitors (TKIs) had been in Phase I/II and III trials [32]. In our study, *CYP3A5* was down-regulated in the drug metabolism pathway. *CYP3A5* encodes a member of the cytochrome P450 superfamily of enzymes which catalyze many reactions involved in drug metabolism [33]. Meanwhile, Downie and his co-works indicated that *CYP3A5* showed a very significantly enhanced expression in the primary ovarian cancers compared with normal ovary [34]. The result above suggested that Drug metabolism and Tyrosine metabolism were associated with the ovarian cancer, and the decreased expression profile of *CYP3A5* may play an important role in the formation and treatment of ovarian cancer.

In addition, we also used STRING tool to get the PPI relationships of the DEGs and gained the network with 405 nodes and 1224 edges. In the network, VEGFA, CALM1, IRC5, POLD1, AURKA, CDT1, BUB1B were selected as hub nodes as their connectivity degrees > 30.

*VEGFA* encodes a glycosylated mitogen belongs to PDGF/VEGF growth factor family, and specifically acts on endothelial cells and has various effects, including mediating increased vascular permeability, inducing angiogenesis, vasculogenesis and endothelial cell growth, promoting cell migration, and inhibiting apoptosis [35]. It is a major mediator of vascular permeability and angiogenesis [36]. Study also indicated *VEGF*-gene was express in all ovarian cancer and peritoneal biopsies, and it induced ascites in ovarian cancer patients due to increased peritoneal permeability through down-regulating the tight junction protein Claudin 5 in the peritoneal endothelium [37]. Thus, *VEGFA* might be one of the target genes for diagnosing ovarian cancer.

At last, we performed the module analysis of the PPI network. The Module A which contained 30 genes was proved closely associated with ovarian cancer. With the GO analysis, the genes in the Module A were significantly enriched in biological processes such as mitotic cell cycle, cell cycle and nuclear division, which indicated cell cycle of mitosis and nuclear division cycle played important roles in ovarian cancer. From the KEGG pathway analysis of Module C, the pathways were also remarkablely enriched in Cell cycle, which confirmed that the mutations in cell cycle have a difference in ovarian cancer.

However, there are some deficiencies of our study. First, the microarray data is not generated by ourselves but from GEO database. Second, the data downloaded from only one platform were comparatively simplex, so the outcome of DEGs may have a high false positive rate. Therefore, further experimental studies should be carried out based on a larger sample size in order to confirm our results.

## Conclusion

As a result of this preliminary study, we confirmed that the pathogenesis of ovarian cancer were closely associated to the mutations of pathways such p53 signaling pathway, drug metabolism, tyrosine metabolism and cell cycle. Besides, we also indicated genes such as *CCNE1*, *CCNB2*, *CYP3A5* and *VEGFA* might play important roles in ovarian cancer and they were predicted target genes for diagnosing the ovarian cancer.

## Competing interest

We certify that regarding this paper, no actual or potential conflicts of interests exist; the work is original, has not been accepted for publication nor is concurrently under consideration elsewhere, and will not be published elsewhere without the permission of the Editor and that all the authors have contributed directly to the planning, execution or analysis of the work reported or to the writing of the paper.

## Authors’ contributions

LF participated in the design of this study, performed the statistical analysis. BW carried out the study, collected important background information, and drafted the manuscript. LF and BW conceived of this study, and participated in the design and helped to draft the manuscript. All authors read and approved the final manuscript.
